The article "Application of ERCP Procedures in Choledocholithiasis with Duodenal Stenosis Patients" was retracted in 2023. Reasons: signs of a paper mill; compromised peer review; unreliable results or conclusions.

# Application of ERCP Procedures in Choledocholithiasis with Duodenal Stenosis Patients

**DOI:** 10.1155/2022/2662435

**Published:** 2022-05-02

**Authors:** Yuyan Shi, Jinghon Zhong, Jianbo Zhou, Qifeng Song

**Affiliations:** ^1^Department of Gastroenterology, Yuyao People's Hospital, Yuyao, Zhejiang, China; ^2^Department of Anesthesiology, Yuyao People's Hospital, Yuyao, Zhejiang, China

## Abstract

**Objective:**

The treatment of choledocholithiasis with duodenal stenosis is a clinical difficult problem. This study aimed to investigate the efficacy and safety of ERCP via gastroscopy in the treatment of choledocholithiasis and duodenal stenosis.

**Methods:**

From January 2015 to December 2020, 21 patients with choledocholithiasis with duodenal stenosis who underwent ERCP treatment under gastroscopy in our hospital were enrolled. The patients' case characteristics, ERCP status, and complication rate were analyzed.

**Results:**

Among the 21 patients, 17 cases were successful in ERCP, and a total of 29 times ERCPs were performed, with an average of 1.71 times per patient. Among the failures of ERCP, selective deep intubation of common bile duct was unsuccessful in 4 cases. Six patients underwent multiple lithotomies, after the operation, of which 4 patients underwent secondary ERCP lithotomy and 2 patients underwent triple ERCP lithotomy. All patients successfully completed the balloon dilation without serious complications. Two patients developed mild acute pancreatitis after ERCP, and all recovered after medication.

**Conclusion:**

In patients with choledocholithiasis and duodenal stenosis, ERCP treatment by gastroscopy has a higher success rate and does not increase the incidence of complications, but there is a problem of cholecystolithiasis recurrence.

## 1. Introduction

Endoscopic retrograde cholangiopancreatography (ERCP) has been used as an important clinical treatment in terms of removing choledocholithiasis and relieving the obstructive jaundice; this method has the advantages of less trauma, good curative effect, and quick recovery, and its efficacy and safety have been widely recognized [1]. Some patients with duodenal bulb ulcers have had posterior duodenal bulb stenosis at the time of treatment, which can form an ectopic nipple lift opening, resulting in poor bile excretion and choledocholithiasis [2]. Prospective data reveal that 10% of adults will develop symptomatic gallstones over the course of a decade in America, and 10–20% of those have concomitant choledocholithiasis [3]. For patients with choledocholithiasis and duodenal stenosis, duodenoscope is often not available, and the use of gastroscope for ERCP and endoscopic treatment can be used as an alternative [4]. The purpose of this study was to retrospectively analyze 21 patients with choledocholithiasis combined with duodenal stenosis, to evaluate the efficacy of ERCP treatment via gastroscopy, and to explore the experience of diagnosis and treatment.

The article "Application of ERCP Procedures in Choledocholithiasis with Duodenal Stenosis Patients" was retracted in 2023. Reasons: signs of a paper mill; compromised peer review; unreliable results or conclusions.

## 2. Materials and Methods

### 2.1. Participants and Data Collection

From January 2015 to December 2020, a total of 21 patients with choledocholithiasis complicated with duodenal stenosis who underwent ERCP treatment through gastroscopy in Yuyao People's Hospital were enrolled. The average age of the 21 patients was 49.5 ± 12.0 years, including 16 males (76.2%) and 5 females (23.8%). Routine medical history inquiries, physical examinations, and imaging evaluations were performed on the patients. Fasting venous blood was collected for routine blood tests, blood coagulation function, liver and kidney function, electrolytes, and blood amylase tests.

Imaging evaluation was performed by abdominal color ultrasound and enhanced CT or MRCP of the upper abdomen. In typical patients, different degrees of dilation, gas accumulation, and filling defects of the intrahepatic and extrahepatic bile ducts can be seen. The patients with choledocholithiasis and duodenal stenosis were diagnosed by symptoms and signs of abdominal pain, elevated ALT, AST, and bilirubin, as well as typical imaging. The patients or their authorized family members have signed an informed consent form. The research plan has been approved by the Ethical Review Committee of Yuyao People's Hospital (YY-2015-012).

### 2.2. Surgical Procedure

Before operation, 10 ml lidocaine mortar was given orally, followed by intramuscular injection of anisodamine 10 mg, diazepam 10 mg, and pethidine 60 mg. The main backup equipment included the Japanese Olympus 260 electronic gastroscope, Boson's yellow zebra guide wire, Poco GIE three-stage expansion balloon, nipple incision, angiography catheter, stone extraction balloon, nasobiliary drainage tube, and biliary plastic stent. The patient was placed in the prone position, oxygen inhalation and ECG monitoring are performed, a transparent cap was installed before the gastroscope, and the endoscope passed through the duodenal stenosis. If necessary, a cylindrical balloon with a diameter of 1.2–1.5 cm was expanded. According to the patient's tolerance, the maximum duration of dilation should not exceed 1 minute. After dilation, selective choledochal intubation angiography was performed to understand the condition of stones in the bile duct. Because of the special position of the nipple opening, a stone extraction balloon or a guidewire basket was used to remove the stone. For patients with incomplete stone removal at one time, multiple stone removals or placed the nasobiliary ducts were given to drain bile. For the recurrence of choledocholithiasis, ERCP was taken again. Routine fasting after surgery, intravenous nutrition, antiinfection, and somatostatin pumping treatment were given. Patients' vital signs and abdominal symptoms and signs were monitored, and bile drainage volume and shape were recorded. The blood amylase was rechecked 2–4 hours postoperatively and the next morning.

The article "Application of ERCP Procedures in Choledocholithiasis with Duodenal Stenosis Patients" was retracted in 2023. Reasons: signs of a paper mill; compromised peer review; unreliable results or conclusions.

Successful selective common bile duct intubation and complete stone removal or partial stone removal + nasobiliary drainage were defined as ERCP success, and failure to find the duodenal papilla or unsuccessful intubation was defined as ERCP failure.

### 2.3. Statistical Analysis

The continuous variable with normal distribution was expressed as mean ± standard deviation, and the categorical variable was expressed by frequency (rate), and statistical analysis was performed using IBM SPSS 21.0 statistical software.

## 3. Results

Table 1 provides the clinical characteristics of the included patients. The mean BMI of 21 patients was 25.7 ± 3.4 kg/m^2^. The number of people with a history of hypertension, coronary heart disease, and diabetes was 5 (23.8%), 3 (14.3%), and 4 (19.0%), respectively. The mean values of alanine aminotransferase and aspartate aminotransferase were 36.8 ± 20.6 U/L and 34.9 ± 23.4 U/L, respectively. The mean values of total bilirubin and direct bilirubin were 12.9 ± 10.2 *μ*mol/L and 6.2 ± 5.3 *μ*mol/L, respectively. The average value of serum amylase was 66.2 ± 47.7 U/L.

As given in Table 2, the disease course of the 21 patients ranged from 1 day to 20 months, and their ages ranged from 29 to 68 years. Among the 21 patients, 17 cases were successful in ERCP, and a total of 29 times ERCPs were performed, with an average of 1.71 times per patient. Among the failures of ERCP, selective deep intubation of common bile duct was unsuccessful in 4 cases. Six patients underwent multiple lithotomies, after the operation, of which 4 patients underwent secondary ERCP lithotomy and 2 patients underwent triple ERCP lithotomy. All patients successfully completed the balloon dilation without serious complications. Two patients developed acute pancreatitis after ERCP, and all recovered after medication.

## 4. Discussion

In this study, we found that among 21 patients with choledocholithiasis complicated with duodenal stenosis, the success rate of ERCP by gastroscopy was 81.0% (17/21), and the average ERCP was 1.71 times per patient. In addition, the incidence of postoperative pancreatitis of ERCP was 9.5% (2/21), and all of them were mild and could get better after drug treatment. ERCP was characterized by a high success rate and few postoperative side effects.

The article "Application of ERCP Procedures in Choledocholithiasis with Duodenal Stenosis Patients" was retracted in 2023. Reasons: signs of a paper mill; compromised peer review; unreliable results or conclusions.

The clinical cases of choledocholithiasis complicated with benign stenosis of the duodenum are relatively rare, and surgical surgery is routinely used for treatment. Some patients may consider endoscopic treatment due to factors such as poor physique, intolerance, or unwillingness to surgery [5]. Combined with this study, we found that routine ERCP is difficult in these patients, and there are problems of recurrence after surgery, and multiple endoscopic treatments are often required. Therefore, the following factors should be paid attention to when ERCP is performed in these patients.

If the patients with choledocholithiasis accompanied by stenosis can be clearly diagnosed before ERCP, it is not necessary to perform duodenoscopy, and the gastroscope with transparent cap can be used directly for the diagnosis and treatment of the patients. A recent study suggested that scar stenosis formed by duodenal bulb ulcers often makes it difficult for duodenoscope to pass the stenosis or increases the risk of duodenal perforation [6]. At this time, the use of a gastroscope with a relatively small diameter may make it easier to pass through the stenosis and reduce the risk of duodenal perforation. Based on the patients' medical history and laboratory examinations, combined with the typical features of bile duct dilatation and filling defect on imaging, the diagnosis can be basically confirmed, and ERCP can be performed directly through gastroscopy.

Balloon dilation is often required before intubation of the common bile duct. Previous studies have suggested that due to bulb ulcers and other reasons, the patients' duodenal bulb scar is deformed, so it is necessary to choose a balloon for expansion to facilitate endoscopic passage [7]. However, the patients' tolerance need to be considered during the expansion process, and some patients may experience severe pain, which may even affect the subsequent operation process [8]. Judging from this group of cases, most of the patients can tolerate well and cooperate to complete the operation. However, in some case groups, local oozing may occur after dilation, and the visual field is poor, and norepinephrine saline is needed for hemostasis.

Previous studies have suggested that the use of a transparent cap gastroscope for ERCP can help to find displaced and deformed duodenal papillae, as well as stone removal treatment [9]. During the use of gastroscopy with transparent cap which can push against the mucous membrane in this group of patients, it was found that the transparent cap could push mucosa, and at the same time, the attraction button was used at the suspicious nipple opening position, which was conducive to the discovery of ectopic nipple opening. However, due to the small operating space in the narrow section behind the ball, the treatment of lithotomy is difficult, and the stone can only be removed with a guidewire basket or a stone extraction balloon.

The article "Application of ERCP Procedures in Choledocholithiasis with Duodenal Stenosis Patients" was retracted in 2023. Reasons: signs of a paper mill; compromised peer review; unreliable results or conclusions.

The recurrence of choledocholithiasis after ERCP lithotomy requires attention. After ERCP, most patients can get choledocholithiasis, but due to unsolved duodenal stenosis, obstructed bile excretion can be caused and recurrent stones are easy [10]. For such patients with repeated recurrences, biliary plastic stents can be placed to improve bile drainage, which may be one of the methods to prevent recurrence of stones [11]. In addition, biliary-enteric anastomosis can also be performed surgically to solve the problem of poor bile excretion. Common bile duct stones after surgery are generally not easy to recur.

Regarding the problem of postoperative pancreatitis, in this study, the incidence of postoperative pancreatitis was 9.5%. In this study, some patients had undergone balloon dilatation, but the incidence of postoperative pancreatitis was basically the same as previous reports, and there was no significant increase [12]. In addition, the 2 cases of postoperative pancreatitis in this study were able to recover and improve after conventional drug treatment without serious complications.

In short, the treatment of choledocholithiasis combined with duodenal stenosis is a clinically urgent problem. Combined with the analysis of this study, we found that balloon dilation of the narrowed duodenum first, followed by ERCP with a transparent cap gastroscope or direct gastroscope, can achieve a higher effect of lithotomy without increasing the incidence of complications. However, it should be noted that there is still a problem of high stone recurrence rate.

## Figures and Tables

**Table 1:** Clinical characteristics of patients.

	Patient population, *n* = 21
Age, years	49.5 ± 12.0
Proportion of males, *n* (%)	16 (76.2)
Duration of disease, days	25 (10, 19)
BMI (kg/m^2^)	25.7 ± 3.4
History of hypertension, *n* (%)	5 (23.8)
History of coronary heart disease, *n* (%)	3 (14.3)
History of diabetes, *n* (%)	4 (19.0)
Alanine aminotransferase (U/L)	36.8 ± 20.6
Aspartate aminotransferase (U/L)	34.9 ± 23.4
Alkaline phosphatase (U/L)	48.3 ± 19.5
Total bilirubin (*μ*mol/L)	12.9 ± 10.2
Direct bilirubin (*μ*mol/L)	6.2 ± 5.3
Blood amylase (U/L)	66.2 ± 47.7

**Table 2:** ERCP of 21 cases of choledocholithiasis with benign stenosis of the duodenum.

No.	Gender	Age	Years ofdisease	Dilationballoondiameter (cm)	Types of treatment endoscopy	Nipple opening	Intubationsituation	Number oflithotomytreatments	Complications
1	Male	45	10 months	1.5	Gastroscope with transparent cap	The back of the ball is near the front wall	Fail	1	None
2	Male	40	20 months	1.4	Gastroscope with transparent cap	Near the big turn after the ball	Fail	1	None
3	Female	39	2 weeks	1.4	Gastroscope with transparent cap	Near the big turn after the ball	Success	2	None
4	Female	59	10 days	1.4	Gastroscope with transparent cap	The back of the ball is near the front wall	Success	1	None
5	Male	68	18 days	1.4	Gastroscope	The back of the ball is near the front wall	Success	1	Pancreatitis
6	Male	62	25 days	1.5	Gastroscope with transparent cap	The back of the ball is near the front wall	Success	1	None
7	Male	39	70 days	—	Gastroscope with transparent cap	The back of the ball is near the front wall	Success	1	None
8	Male	44	3 months	—	Gastroscope with transparent cap	Near the big turn after the ball	Success	3	None
9	Female	57	7 months	—	Gastroscope with transparent cap	Near the big turn after the ball	Success	2	None
10	Male	61	1 week	—	Gastroscope with transparent cap	Near the big turn after the ball	Fail	1	Pancreatitis
11	Male	31	20 days	1.4	Gastroscope	The back of the ball is near the front wall	Success	1	None
12	Female	40	1 year	—	Gastroscope with transparent cap	The back of the ball is near the front wall	Fail	1	None
13	Male	29	6 months	1.2	Gastroscope with transparent cap	Cannot peek	Success	1	None
14	Male	59	10 days	—	Gastroscope with transparent cap	Near the big turn after the ball	Success	2	None
15	Male	67	3 days	—	Gastroscope with transparent cap	The back of the ball is near the front wall	Success	1	None
16	Male	55	1 day	—	Gastroscope with transparent cap	The back of the ball is near the front wall	Success	3	None
17	Male	37	15 days	—	Gastroscope with transparent cap	Near the big turn after the ball	Success	1	None
18	Female	42	1 month	1.4	Gastroscope with transparent cap	Near the big turn after the ball	Success	1	None
19	Male	56	3 months	1.5	Gastroscope	The back of the ball is near the front wall	Success	1	None
20	Male	63	10 months	—	Gastroscope with transparent cap	The back of the ball is near the front wall	Success	2	None
21	Male	47	1 day	—	Gastroscope with transparent cap	The back of the ball is near the front wall	Success	1	None

The article "Application of ERCP Procedures in Choledocholithiasis with Duodenal Stenosis Patients" was retracted in 2023. Reasons: signs of a paper mill; compromised peer review; unreliable results or conclusions.

## Data Availability

The data used to support the findings of this study are available from the corresponding author upon request.
